# Feature Point Extraction and Motion Tracking of Cardiac Color Ultrasound under Improved Lucas–Kanade Algorithm

**DOI:** 10.1155/2021/4959727

**Published:** 2021-08-03

**Authors:** Xiaoli Zhang, Punan Li, Yibing Li

**Affiliations:** ^1^Department of Ultrasound Medicine, Jincheng People's Hospital, Jincheng, Shanxi 048000, China; ^2^Department of Ultrasound Medicine, Zhengzhou Maternity Hospital Affiliated to Henan University, Zhengzhou, Henan 450000, China

## Abstract

The purpose of this research is to study the application effect of Lucas–Kanade algorithm in right ventricular color Doppler ultrasound feature point extraction and motion tracking under the condition of scale invariant feature transform (SIFT). This study took the right ventricle as an example to analyze the extraction effect and calculation rate of SIFT algorithm and improved Lucas–Kanade algorithm. It was found that the calculation time before and after noise removal by the SIFT algorithm was 0.49 s and 0.46 s, respectively, and the number of extracted feature points was 703 and 698, respectively. The number of feature points extracted by the SIFT algorithm and the calculation time were significantly better than those of other algorithms (*P* < 0.01). The mean logarithm of the matching points of the SIFT algorithm for order matching and reverse order matching was 20.54 and 20.46, respectively. The calculation time and the number of feature points for the SIFT speckle tracking method were 1198.85 s and 81, respectively, and those of the optical flow method were 3274.19 s and 80, respectively. The calculation time of the SIFT speckle tracking method was significantly lower than that of the optical flow method (*P* < 0.05), and there was no statistical difference in the number of feature points between the SIFT speckle tracking method and the optical flow method (*P* > 0.05). In conclusion, the improved Lucas–Kanade algorithm based on SIFT significantly improves the accuracy of feature extraction and motion tracking of color Doppler ultrasound, which shows the value of the algorithm in the clinical application of color Doppler ultrasound.

## 1. Introduction

Commonly used imaging techniques for evaluating cardiac tissue function include Doppler tissue imaging, magnetic resonance imaging (MRI), computerized tomography (CT), and ultrasound. Ultrasound imaging is widely used in the evaluation of cardiac tissue function due to its advantages of fast imaging speed, high safety, and low price [1]. At present, the evaluation of cardiac function by clinical diagnostic technology is mainly the evaluation of left ventricular function, and the research of right ventricle is still relatively vacant in the medical field. The change of right ventricular function is of great significance for the evaluation, diagnosis, and prognosis of pulmonary hypertension and a variety of heart diseases [2]. Cardiac color Doppler ultrasound is the main examination method in the clinical diagnosis of CHF, and it is also the only imaging method that can display the internal structure of the heart and internal circulation of organs. This method is simple to operate, has no wound, and can carry out repeated operation. When examining patients with CHF, it can display the cardiac image structure comprehensively and intuitively, Therefore, cardiac color Doppler ultrasound can accurately and comprehensively evaluate the function of right ventricle and myocardium, which plays an important role in the diagnosis and treatment of heart disease [3]. Due to the randomness of ultrasound scattering signals in biological tissues, a large amount of irregular speckle noise will be distributed in the generated image, which will make the image blurred, and the artifacts of different organs will also affect the ultrasound imaging [4]. The acoustic field characteristics of the ultrasound beam make the lateral resolution of ultrasound imaging low. Ordinary ultrasound images usually cannot clearly reflect the tissue morphology and differences between tissues [5]. The complexity of the geometry leads to the lack of accurate measurement of right ventricular function by ultrasound inspection methods [6].

The optical flow method can process continuous image sequences and has real-time characteristics in digital image data. Lucas–Kanade algorithm is an optical flow estimation algorithm based on two-frame difference. Lucas–Kanade point matching algorithm has a wide range of applications in realizing single and multiple target tracking because of its fast calculation speed and simple application [6]. However, the tracking effect of Lucas–Kanade algorithm in practice is not good [7]. Some researchers proposed that the idea of image pyramids can be introduced into the Lucas–Kanade algorithm, which can significantly increase its tracking effect [8]. There were studies applying the Lucas–Kanade algorithm to the motion tracking of cardiac color Doppler ultrasound. However, the effect of feature point extraction and tracking is still poor when the motion between frames of the sequence image is large, because the Lucas–Kanade algorithm uses linear estimation [6], and further optimization is needed.

In summary, although Lucas–Kanade algorithm has significant advantages in target tracking, it still needs further improvement in cardiac color Doppler ultrasound feature point extraction and motion tracking. Therefore, the idea of pyramid was proposed based on the Lucas–Kanade algorithm and the SIFT algorithm to improve the accuracy and computing speed of the Lucas–Kanade algorithm, which was applied to the right ventricular color Doppler ultrasound feature point extraction and motion tracking. It was hoped that this research can provide a reference basis for the evaluation, diagnosis, and prognosis of pulmonary hypertension and a variety of heart diseases.

## 2. Materials and Methods

### 2.1. Lucas–Kanade Algorithm Improvement

Differentiation method [9] and region-based matching method [10] are the most commonly used algorithms for optical flow algorithms, and Lucas–Kanade algorithm is an algorithm based on the local constraints of optical flow. For the small plane *S* with the center line *A*, the gray values of the pixels in the regional coordinates of any two images in the image sequence are *F*(*x*) and *G*(*x*), respectively. Then, the smallest difference between the two images is expressed as shown in equation (1), where *b* is the vector for calculating the matching.

(1) $$\begin{array}{c} D=\sum_{x\in S}\left|F\left(x+b\right)-G\left(x\right)\right|. \end{array}$$

If *b*⟶0, then there the following equations:

(2) $$\begin{array}{c} F\left(x\right)\approx \frac{F\left(x+b\right)-F\left(x\right)}{b}=\frac{G\left(x\right)-F\left(x\right)}{F\left(x\right)},\\ b\approx \frac{G\left(x\right)-F\left(x\right)}{F\left(x\right)}. \end{array}$$

The weight of *b* obtained at the *x* field is expressed as follows:

(3) $$\begin{array}{c} w\left(x\right)=\frac{1}{\left|G\left(x\right)-F\left(x\right)\right|}. \end{array}$$

The iterative equation of the matched vector *b* is expressed as equation (4), where *k* is the number of iterations.

(4) $$\begin{array}{c} b_{k+1}=b_{k}+\frac{\sum_{x}\left(\left(w\left(x\right)\left[G\left(x\right)-F\left(x+b_{k}\right)\right]\right)/\left(F\left(x+b_{k}\right)\right)\right)}{\sum_{x}w\left(x\right)}. \end{array}$$

For the accuracy and speed of the Lucas–Kanade algorithm, the pyramid idea was introduced into the Lucas–Kanade algorithm to iterate the Lucas–Kanade algorithm by levels and reduce the calculation amount of Lucas–Kanade algorithm caused by excessive image pixel motion [11]. For the point (*x*, *y*) on the ultrasound image, the iterative equation of the improved Lucas–Kanade algorithm based on the pyramid idea is expressed as follows:

(5) $$\begin{array}{c} C^{l}=\frac{1}{4}\left(2x,2y\right)+\frac{1}{8}\left[C^{l-1}\left(2x-1,2y\right)+C^{l-1}\left(2x+1,2y\right)+C^{l-1}\left(2x,2y-1\right)+C^{l-1}\left(2x,2y+1\right)\right]+16\left[C^{l-1}\left(2x-1,2y-1\right)+C^{l-1}\left(2x-1,2y+1\right)+C^{l-1}\left(2x+1,2y-1\right)+C^{l-1}\left(2x+1,2y+1\right)\right]. \end{array}$$

In equation (6), *C*^*l*−1^() is the gray value of the point (*x*, *y*) at time *l*.

As the number of pyramid layers progresses downwards, the resolution of the image gradually decreases. The optical flow field motion result obtained in the image of the previous resolution will be used as the initial value for the calculation of the next resolution. Calculating the Lucas–Kanade algorithm in a hierarchical manner can greatly reduce the massive data calculations generated when a large amount of optical flow moves and shortens the calculation time. The iterations were repeated until the final optical flow result was calculated. The schematic diagram of the improved operation of the Lucas–Kanade algorithm pyramid is shown in Figure 1.

### 2.2. Ultrasonic Image Preprocessing

The ultrasound imaging system will cause the image to be damaged to a certain extent during image acquisition, transmission, and preservation. Therefore, it is necessary to perform operations such as line filtering noise on the cardiac color Doppler ultrasound image to reduce the impact on the image before the data analysis on cardiac color Doppler ultrasound. Commonly used medical image noise reduction methods include mean filter, adaptive Wiener filter, and median filter [12]. The linear-mean filtering method filters out isolated noise points by means of averaging neighborhoods and has a good removal effect on salt and pepper noise, Gaussian noise, and impulse noise [13]. For the image pixel point (*x*, *y*) to be filtered, the corresponding *R* of the linear-mean filtering is expressed as follows:

(6) $$\begin{array}{c} R=w\left(-1,-1\right)f\left(x-1,y-1\right)+w\left(-1,0\right)f\left(x-1,y\right)+w\left(0,0\right)f\left(x,y\right)+\cdots +w\left(1,0\right)f\left(x+1,y\right)+w\left(1,1\right)f\left(x+1,y+1\right). \end{array}$$

On the image *g* with a mask size of *M* × *N*, the filter mask of linear-mean filtering is *m* × *n*, and the corresponding pixel is expressed as follows:

(7) $$\begin{array}{c} f\left(x,y\right)=\frac{1}{D}\sum_{\left(x,y\right)\in N}g\left(x,y\right). \end{array}$$

D represents the sum of pixels in the mask including the current pixel, and *g*(*x*, *y*) is the pixel value in the *x*-th row and *y*-column.

### 2.3. Feature Points Extraction of Cardiac Ultrasound Images

Ultrasound image speckle is a feature often used in medical ultrasound image processing. The feature speckles of cardiac ultrasound images usually reflect changes in the heart cavity, myocardium, and valves during movement. Forstner algorithm, SUNSAN algorithm, SIFT algorithm, and Harris algorithm are commonly used point feature extraction methods in the field of image registration. Among them, the SIFT algorithm has the characteristics of strong matching ability, stable extraction of features, and high matching accuracy. It can also match features between two images with large differences [14]. Gaussian normal distribution function *G*(*x*, *y*, *σ*) of the SIFT algorithm in a two-dimensional plane image is expressed as follows:

(8) $$\begin{array}{c} G\left(x,y,\sigma \right)=\frac{1^{e-\left(x2+y2\right)/2\sigma^{2}}}{2\pi \sigma^{2}}. \end{array}$$

Its scale space is expressed as follows:

(9) $$\begin{array}{c} L\left(x,y,\sigma \right)=G\left(x,y,\sigma \right)*I\left(x,y\right). \end{array}$$

In equations (8) and (9), (*x*, *y*) is the position of a certain pixel of the target image, *L*(*x*, *y*, *σ*) is the scale space of the target image, and *σ* is the scale coordinate. *σ* is related to the smoothness of the image. The smaller the *σ*, the lower the smoothness. The calculation of Gaussian difference scale space is as follows:

(10) $$\begin{array}{c} D\left(x,y,\sigma \right)=\left[G\left(x,y,k\sigma \right)-G\left(x,y,\sigma \right)\right]*I\left(x,y\right)=L\left(x,y,k\sigma \right)-L\left(x,y,\sigma \right). \end{array}$$

A fitted quadratic function was used to increase the accuracy of the position detection of the feature point. For the key points and boundary points with insignificant features in the extraction process, the spatial scale function was used to eliminate the algorithm to enhance the robustness and accuracy of the algorithm. The spatial scale function is expressed as follows:

(11) $$\begin{array}{c} D\left(x,y,\sigma \right)=D\left(x,y,\sigma \right)+\left(\frac{\partial D^{t}}{\partial x}+\frac{1}{2}x^{t}\frac{\partial^{2}D}{\partial x^{2}}x\right). \end{array}$$

Derivation of the above function is the calculation method of accurate position.

(12) $$\begin{array}{c} \hat{x}=-{\frac{\partial^{2}D^{-1}}{\partial x^{2}}}^{t}\frac{\partial D}{\partial x}. \end{array}$$

The key points with insignificant features are eliminated, and the following equation is obtained.

(13) $$\begin{array}{c} D\left(\hat{x}\right)=D\left(x,y,\sigma \right)+\frac{1}{2}x\frac{\partial D^{t}}{\partial x}, \end{array}$$

$\hat{x}$ is the transpose of the matrix (*x*, *y*, *σ*). If $D\left(\hat{x}\right)\geq 0.03$, the feature point is retained; otherwise, it is discarded.

SIFT algorithm makes use of the gradient direction distribution characteristics of neighborhood pixels of key points to specify direction parameters for each key point, so that the operator has rotation invariance [15].

(14) $$\begin{array}{c} m\left(x,y\right)=\sqrt{{\left[L\left(x+1,y\right)-L\left(x-1,y\right)\right]}^{2}+{\left[L\left(x,y+1\right)-L\left(x,y-1\right)\right]}^{2}}, \end{array}$$

(15) $$\begin{array}{c} \vartheta \left(x,y\right)=\alpha \;\tan\;2\left[\frac{L\left(x+1,y\right)-L\left(x-1,y\right)}{L\left(x,y+1\right)-L\left(x,y-1\right)}\right]. \end{array}$$

In equations (15) and (16), *m*(*x*, *y*) is the calculation equation for gradient modulus at position (*x*, *y*), and *δ*(*x*, *y*) is the calculation equation for Angle at position (*x*, *y*). *L* is the scale space.

The required calculation method of the circular image area in the process of generating the features of key points is as follows:

(16) $$\begin{array}{c} R=\frac{3\sqrt{2}\sigma \left(d+1\right)+1}{2}. \end{array}$$

The coordinate of rotation Angle obtained after movement is expressed as follows:

(17) $$\begin{array}{c} \left[\begin{array}{c} \hat{x}\\ \hat{y} \end{array}\right]=\left[\begin{array}{c} \cos\;\alpha -\sin\;\alpha \\ \cos\;\alpha +\sin\;\alpha \end{array}\right]\times \left[\begin{array}{c} x\\ y \end{array}\right], \end{array}$$

In equations (16) and (17), *σ* is the intragroup scale of the group, where the feature points are located, and *α* is the rotation Angle.

The calculation method of specification description subvector element is as follows:

(18) $$\begin{array}{c} l_{j}=\frac{w_{j}}{\sqrt{\sum_{i=1}^{128}w_{i}}}, \end{array}$$

*w*_*i*_ and *w*_*j*_ are eigenvectors of *i* and *j* dimensions, and *l*_*i*_ is normalized vector.

The extraction steps of feature points in cardiac ultrasound images based on SIFT algorithm mainly included five parts: generation of scale space, detection of extreme points in scale space, accurate positioning of extreme points, direction parameters of key points, and generation of feature vectors of key points. The specific SIFT algorithm feature point extraction flow chart is shown in Figure 2.

### 2.4. Feature Point Matching and Tracking Based on Improved Lucas–Kanade Algorithm

Euclidean distance is often used to verify whether the feature points of two images match [16]. It is assumed that the two images to be matched are A and B, and SIFT is used to extract feature points for the two images. If *f*_*a*_={*a*_1_, *a*_2_,…, *a*_*m*_} and *f*_*b*_={*b*_1_, *b*_2_,…, *b*_*m*_} are the feature point sets of *A* and *B*, respectively, and *m* and *n* are the number of feature points of *A* and *B*, respectively, then the Euclidean distance of *k*-dimensional space is expressed as follows:

(19) $$\begin{array}{c} s\left(f_{a},f_{b}\right)=\text{sqrt}\left[\sum_{i=1}^{k}{\left(a_{i}-b_{i}\right)}^{2}\right]. \end{array}$$

For a certain point, the Euclidean distance in *f*_*a*_ and *f*_*b*_ was calculated to find the minimum distance and the second smallest distance $\tilde{d_{\min}}$, $r=d_{\min}/\tilde{d_{\min}}$. Whether the feature points are matched is evaluated according to the following equation, where evaluation is the threshold set by the experiment, which was set as 0.44 in this research.

(20) $$\begin{array}{c} \left\{\begin{array}{cc} r<\eta , & \text{success,}\\ r\geq \eta , & \text{failure.} \end{array}\right. \end{array}$$

K-D tree index tree and Best Bin First (BBF) algorithm are commonly used in feature point matching process. BBF algorithm reduces the node backtracking of K-D tree nearest neighbor search algorithm, improves the search efficiency, and is suitable for high-dimensional data search. For two images to be matched, feature points extraction and feature vector set analysis were carried out by SIFT, and the corresponding point set of SIFT feature matching was finally obtained. The flowchart of feature point matching based on the improved Lucas–Kanade algorithm is shown in Figure 3.

### 2.5. Statistical Methods

The experimental data was processed using SPSS 19.0, the count data was tested by *χ*^2^ test, and *P* < 0.05 indicated that the difference was statistically considerable.

## 3. Results and Discussion

### 3.1. Image Motion Feature Point Detection Based on Improved Lucas–Kanade Algorithm

The image sequence of frames 1 to 2 of the right ventricular movement cycle was selected for comparative analysis, and the vector image of gray-scale movement from frame 1 to frame 2 was obtained. The results are shown in Figure 4. It can be concluded from Figure 4(c) that the improved Lucas–Kanade algorithm has better real-time performance in feature point tracking. The gradient direction histogram of Lucas–Kanade algorithm represented the gradient direction and the total number of gradients. Gradient direction histogram was used to obtain the direction synthesis vector of an image pixel in a certain area. The reference direction was calculated through the small area, where the key points were obtained, so that the algorithm had spatial rotation invariance [17].

### 3.2. Special Point Trajectory Based on Improved Lucas–Kanade Algorithm

The improved Lucas–Kanade algorithm was used to compare the movement tracks of right ventricular myocardium, right atrioventricular septal tricuspid valve ring, and left atrioventricular septal tricuspid valve ring (Figure 5). The motion trajectory of feature points based on the improved Lucas–Kanade algorithm had significant differences for different parts. The variation range of the right ventricular myocardium in the *X* direction was 372∼405, and the variation range of the right atrioventricular septal tricuspid valve in the *X* direction was 385∼450. The left ring of the atrioventricular septal tricuspid valve varied from 415 to 450 in the *X* direction. Heart movement is a very complex nonlinear movement, which includes rotation, torsion, and circular movement, in addition to contraction and diastole, and the motion parameters of each point and region are often different [18].

### 3.3. Analysis of Feature Point Extraction Results Based on Improved Lucas–Kanade Algorithm

The improved Lucas–Kanade algorithm was used to extract ultrasonic images with feature points, and the number of feature points under different image frame sequences was statistically analyzed (Figure 6). The number of feature points extracted under different image frame order had great difference. When the image frame order was 1, the maximum number of feature points extracted was 75.

The calculation time and the number of feature points of different algorithms before and after noise removal were compared (Figure 7). The calculation time of SIFT algorithm before noise removal was 0.49 s, and the calculation time of Forstner, SUNSAN, and Harris was 1.71 s, 3.04 s, and 2.25 s, respectively. The calculation time of SIFT algorithm after noise removal was 0.46 s, and the calculation time of Forstner, SUNSAN, and Harris was 1.12 s, 2.89 s, and 2.11 s, respectively. The calculation time of the SIFT algorithm before and after the noise was removed was obviously shorter than that of other algorithms. The calculation time of all algorithms after noise removal was significantly shorter than that before noise removal. The number of feature points extracted by the SIFT algorithm before noise removal was 703, and the number of feature points extracted by the Forstner, SUNSAN, and Harris algorithms was 182, 426, and 535, respectively. The number of feature points extracted by the SIFT algorithm after noise removal was 698, and the number of feature points extracted by the Forstner, SUNSAN, and Harris algorithms was 126, 76, and 228, respectively. The number of feature points extracted by SIFT algorithm before and after noise removal was more than that of other algorithms, and the number of feature points extracted by all algorithms after noise removal was significantly less than that before noise removal. It showed that, among the four feature point extraction algorithms, the SIFT algorithm extracted the largest number of speckles and took the least time. The number of feature points extracted by the SIFT algorithm and the calculation time were significantly better than those of other algorithms (*P* < 0.01).

The different algorithms before and after noise removal were compared on the first frame of the heart motion image to extract the feature point images (Figure 8). Different algorithms had large differences in the number of feature points extracted from the diastolic motion image of the short-axis motion of the left ventricle with a size of 172 × 172. The speckles extracted by the Forstner operator were more uniformly dispersed, but the number of extracted feature points was small. Although SUNSAN and Harris algorithms extracted more features than Forstner operators, their calculation time was longer. The number of feature extraction points of SIFT algorithm was obviously more than that of other algorithms. Forstner operator was the best method for feature points compared with the other three methods.

### 3.4. Analysis of Feature Point Matching Results Based on Improved Lucas–Kanade Algorithm

To test the accuracy of the SIFT algorithm, the ultrasound images of the first and second frames of the same heart were matched, and the results were shown in Figure 9. By observing the distribution of red spots in the image, it can be concluded that sift algorithm has good stability and accuracy.

To further objectively analyze the accuracy of the feature point matching of the SIFT algorithm, the order matching method and the reverse order matching method were used to extract the matching point logarithms under different frame sequences (Figure 10(a)). The logarithm of the matching points extracted by the sequential matching method and the reverse matching method was not much different. The mean logarithm of the matching points of the sequential matching method and the reverse matching method was 20.54 and 20.46, respectively, which indicated that, for the same two sets of images, the matching algorithm can be used as a template for each other, which had little effect. The matching results of different ultrasonic image feature extraction points were compared (Figure 10(b)). When the image frame order was 5–11, the feature extraction point matching effect was ideal.

### 3.5. Analysis of Feature Point Tracking Results Based on Improved Lucas–Kanade Algorithm

Based on the characteristics of two-dimensional speckle tracking in ultrasonic image, the tolerance method was selected to track the image sequence. The selected feature points were modified within 1∼20 pixels, and a point (130,165) on the myocardial interval between the left and right ventricles was selected for tracking under different tolerance conditions. The tracking results of the first 30 frames of the ultrasonic image sequence were shown in Table 1 and Figure 11. Feature points were extracted in both the 6th and 7th frames. The reason may be that the sequences of matching points between two adjacent frames are not identical, leading to the occurrence of missing matching [19].

### 3.6. Comparison of Tracking Results of Feature Points by Different Algorithms

The shrinkage of feature points per frame of SIFT speckle tracking method and optical flow method was compared (Figure 12). The highest point and curvature of SIFT speckle tracking method were close to the original curve, while the highest point and curvature of optical flow method were different from the original curve. The differences between the two methods were analyzed. The possible reason was that the intraregion matching of SIFT speckle tracking method improved the accuracy of matching, while optical flow tracking in the neighborhood of key points was less affected by noise and had good stability, but its accuracy was low [20].

The calculation time and number of tracking speckles of SIFT speckle tracking method and optical flow method were compared (Figure 13). The calculation time and number of tracking speckles of SIFT speckle tracking method were 1198.85 s and 81, respectively, and the calculation time and number of tracking speckles of optical flow method were 3274.19 s and 80, respectively. The calculation time of SIFT speckle tracking method was significantly lower than that of optical flow method, and the difference between them was great (*P* < 0.05). There was no remarkable difference in the number of tracking speckles between SIFT and optical flow method (*P* > 0.05).

The above results show that Lucas–Kanade algorithm improved by pyramid idea, SIFT algorithm, and denoising algorithm is superior to other algorithms in terms of calculation time, number of feature points identified, and number of tracking spots. Yang et al. [21] used the improved ROAM algorithm based on pyramid idea to preprocess large amount of terrain and texture data in layers and blocks and obtained the conclusion combined with the algorithm, the 3D terrain of Huairou Reservoir in Beijing was rendered, and the real-time network roaming was carried out. Liu et al. [22] also studied the defect image registration based on SIFT algorithm and found that the algorithm can effectively register the defect image and lay a good foundation for the subsequent defect information extraction. The above research results show that the application effect of pyramid idea and sift algorithm is basically consistent with this research. However, Lv et al. [23] used the pyramid Lucas–Kanade combined with U-net technology to study its matching performance on renal free breathing multi-b-value diffusion MRI and obtained the segmentation based on U-net and pyramid Lucas–Kanade registration method, so as to improve the alignment of multi-b-value diffusion weighted MRI and reduce the interference in free breathing.

## 4. Conclusion

The application value of the improved Lucas–Kanade algorithm based on SIFT in the extraction of feature points and motion tracking of heart color ultrasound was discussed. Pyramid idea, SIFT algorithm, and noise reduction algorithm were introduced to improve the Lucas–Kanade algorithm. The results showed that the improved Lucas–Kanade algorithm was better than other algorithms in the computation time, the number of recognized feature points, and the number of tracking speckles. However, there are still some shortcomings in this study. There are mismatching problems in multiple similar regions in the process of speckle tracking. In the future work, the coherence of the feature points of the image sequence will be enhanced according to the image features of the heart color ultrasound, so as to reduce the mismatching phenomenon and further improve the accuracy of the matching of the feature points. In conclusion, the improved Lucas–Kanade algorithm based on SIFT proposed significantly improves the accuracy of feature point extraction and motion tracking of cardiac color ultrasound. It shows that the algorithm has a good prospect in the clinical application of cardiac color Doppler ultrasound.

## Figures and Tables

**Figure 1:** Schematic diagram of pyramid improvement of Lucas–Kanade algorithm.

**Figure 2:** Specific flow chart of feature point extraction of SIFT algorithm.

**Figure 3:** Flow chart of feature point matching based on improved Lucas-Kanade algorithm.

**Figure 4:** Image sequence of frames 1-2 of right ventricular movement cycle. (a) Image of frame 1; (b) Image of frame 2; (c) vector diagram of gray-scale motion.

**Figure 5:** Motion trajectories of special points in optical flow method.

**Figure 6:** Statistics of the number of special points extracted by the SIFT algorithm.

**Figure 7:** Comparison of calculation time and number of feature points before and after noise removal by different algorithms. (a) Comparison of calculation time before and after noise removal by different algorithms; (b) comparison of the number of feature points before and after noise removal by different algorithms. ^*∗*^indicates a remarkable difference compared with SIFT, *P* < 0.01.

**Figure 8:** Analysis of feature point extraction results of different algorithms. (a) Original image; (b) feature point extraction effect of Forstner algorithm; (c) feature point extraction effect of SUNSAN algorithm; (d) feature point extraction effect of Harris algorithm; (e) feature point extraction effect of SIFT algorithm.

**Figure 9:** Matching results of cardiac ultrasound images in frames 1-2.

**Figure 10:** Feature point matching results based on the improved Lucas–Kanade algorithm. (a) Comparison of the results of sequential matching and reverse matching; (b) comparison of matching results of different templates.

**Figure 11:** Spatial displacement of feature point matching based on the improved Lucas–Kanade algorithm.

**Figure 12:** Comparison of shrinkage per frame under different algorithms.

**Figure 13:** Comparison of the number of tracking speckles and calculation time of different algorithms. (a) Comparison of calculation time of different algorithms; (b) comparison of the number of tracking speckles of different algorithms. ^*∗*^indicates remarkable difference versus SIFT, *P* < 0.05.

**Table 1:** Image tracking table for frames 1 to 30.

Point	Abscissa	Ordinate	Point	Abscissa	Ordinate	Point	Abscissa	Ordinate
1	129.17	158.17	11	129.17	108.19	21	124.11	39.17
2	130	141.92	12	131.52	98.49	22	112.98	33.25
3	128	115.54	13	122.68	99.12	23	121.00	33.16
4	110.92	112.68	14	118.45	80.16	24	115.19	39.45
5	121.41	111.54	15	125.14	88.12	25	112.58	38.12
6	0	0	16	112.52	78.16	26	114.16	110.17
7	0	0	17	133.41	75.54	27	124.51	39.54
8	117.41	104.19	18	128.26	67.77	28	112.51	38.77
9	129.16	112.44	19	124.71	41.25	29	114.79	35.75
10	119.28	110.62	20	122.64	51.22	30	120.18	38.16

## Data Availability

The data used to support the findings of this study are available from the corresponding author upon request.
